The article "Chemical Characterization and Antioxidant, Antimicrobial, and Insecticidal Properties of Essential Oil from Mentha pulegium L" was published in 2021. Journal: Evid Based Complement Alternat Med.

# Chemical Characterization and Antioxidant, Antimicrobial, and Insecticidal Properties of Essential Oil from *Mentha pulegium* L.

**DOI:** 10.1155/2021/1108133

**Published:** 2021-10-15

**Authors:** Allali Aimad, Rezouki Sanae, Fadli Anas, El Moussaoui Abdelfattah, Mohammed Bourhia, Ahmad Mohammad Salamatullah, Abdulhakeem Alzahrani, Heba Khalil Alyahya, Nawal A. Albadr, Agour Abdelkrim, Azeddin El Barnossi, Eloutassi Noureddine

**Affiliations:** ^1^Laboratory of Animal and Plant Production, and Agro-Industry, Faculty of Sciences, Ibn Tofail University BP 133, Kenitra 14000, Morocco; ^2^Southwest Florida Research and Agricultural Center, IFAS, University of Florida, Immokalee, FL 34142, USA; ^3^Laboratory of Biotechnology, Environment, Agrifood and Health, Faculty of Science, University of Sidi Mohamed Ben Abdellah, Fez 30050, Morocco; ^4^Laboratory of Chemistry, Biochemistry, Nutrition, and Environment, Faculty of Medicine and Pharmacy, University Hassan II, Casablanca 20000, Morocco; ^5^Department of Food Science & Nutrition, College of Food and Agricultural Sciences, King Saud University, P.O. Box 2460, Riyadh 11451, Saudi Arabia; ^6^Laboratory of Natural Substances, Pharmacology, Environment, Modeling, Health & Quality of Life, Faculty of Sciences, Sidi Mohamed Ben Abdellah University, Fez, Morocco; ^7^Regional Center for the Trades of Education and Training (CRMEF), Fez, Morocco

## Abstract

The chemical composition and antibacterial, insecticidal, and antioxidant properties of the essential oil from *Mentha pulegium* L. (*M. pulegium*) growing in Morocco were investigated in this work. To achieve this goal, the oils were obtained by using hydrodistillation before being characterized by GC-MS. The antibacterial and antifungal activities were conducted against pathogenic strains using the disc diffusion and MICS bioassays. The insecticidal activity was carried out versus *C. maculatus* using contact and inhalation tests. The antioxidant activity was performed by using DPPH and total antioxidant capacity bioassays. The chemical analysis of the oil showed that 20 compounds were identified, which represented 98.91% of the total oil. In the oil, the main components detected were R-(+)-pulegone (76.35%), carvone (5.84%), dihydrocarvone (5.09%), and octanol-3 (2.25%). The essential oil has moderate-to-strong broad-spectrum antibacterial and antifungal properties; the results showed that *B. subtilis* was the most sensitive strain to *M. pulegium* oil, with the largest inhibition diameter (25 ± 0.33). For the antifungal activity, the results obtained indicated that *Aspergillus niger* was the most sensitive fungal strain to *M. pulegium* oil with an inhibition percentage up to 100%. Regarding the insecticidal activity, the inhalation test showed a high efficacy (100% mortality), and a lethal concentration of LC_50_ = 1.41 + 0.48 *μ*L/L air was obtained after 24 hours of exposure. Moreover, the contact test showed that a total reduction in fertility and emergence was obtained with a dose of 20 *μ*L/mL of acetone. Regarding the antioxidant activity, the sample concentration necessary to inhibit 50% of HE radicals (IC_50_) was 7.659 mg/mL (DPPH) and 583.066 57.05 mg EAA/g EO (TAC).

The article "Chemical Characterization and Antioxidant, Antimicrobial, and Insecticidal Properties of Essential Oil from Mentha pulegium L" was published in 2021. Journal: Evid Based Complement Alternat Med.

## 1. Introduction

Morocco's geographical location provides a diverse spectrum of bioclimates, allowing for the formation of diverse flora [1, 2]. The floral wealth is largely related to the ecological heterogeneity of the biotopes. Indeed, it can go from the desert to the high mountains, which allows the development of various species with different bioclimatic stages. The country possesses ancient know-how [3], which has been conserved throughout the ages, in addition to this especially favorable natural setting. In this sense, herbal medicine has witnessed large use by the indigenous people in flavoring and preserving foodstuffs. In Morocco, more than 400 plant species have been accounted for medicinal use [4].

Essential oil (EO) from plants is an important resource of natural products and their components are mainly used as food flavors. Additionally, EO has also non-food applications including antifungal, antimicrobial, antioxidant, and insecticidal activity [5–9]. This confirms the importance of these natural products to develop new alternative solutions in several areas such as health, food safety, and agriculture.

*Mentha pulegium* L. (*M. pulegium*) is an indigenous perennial plant found in Europe, North Africa, and the Middle East [10]. Species among *Mentha* (Labiatae) are widely used against several diseases with a wide spectrum of use, which varies from one region to another. Various research has also revealed that the plant extracts are frequently used as an anti-inflammatory, antispasmodic, carminative, antitussive, diaphoretic, antiemetic, analgesic, stimulant, and emmenagogue and in the form of powders, infusions, and decoctions [11]. The presence of numerous secondary metabolites, including phenolic chemicals, flavonoids, and essential oils, is primarily responsible for these characteristics [12–14].

*M. pulegium* is an important source of essential oils with pharmacological activities including allelopathic properties [15]. In addition, we found that the essential oil of *M. pulegium* leaves exhibited significant insecticidal activity against individuals of *Oryzaephilus surinamensis*, causing a total population reduction at the highest dose [16]. It would be interesting to discover whether *M. pulegium* essential oil and its components have insecticidal properties against other species. As a result, we studied the chemical composition of *M. pulegium* essential oils, as well as their insecticidal activities against *Callosobruchus maculatus*, one of the most common pests of chickpea grains in Morocco along with antioxidant activity, and antimicrobial activity against some pathogenic strains in this study.

The article "Chemical Characterization and Antioxidant, Antimicrobial, and Insecticidal Properties of Essential Oil from Mentha pulegium L" was published in 2021. Journal: Evid Based Complement Alternat Med.

## 2. Material and Methods

### 2.1. Plant Material and Oil Extraction

*M. pulegium* was collected from the Moroccan region of Ouazzane (34°47′49 N, −5°34′56 W). The botanical identification was carried out by a botanist at Sidi Mohamed Ben Abdellah University, where the reference specimen number DM01/02501 was deposited. Thereafter, the aerial part of the plant was dried in the shade in a dry and ventilated area of the laboratory at a temperature between 25 and 32°C. Briefly, 100 g of *M. pulegium* leaves and buds was subjected to essential oil extraction by using hydrodistillation for 3 hours.

### 2.2. GC-MS of Essential Oils

The identification of the essential oil composition was carried out by gas chromatography-mass spectrometry (GC-MS). Analysis was performed using GC system with a flame ionization detector and an HP-5MS capillary column. Temperature programmed gas chromatography was set to 35°C and 250°C with a gradient of 5°C/min. Gas chromatography with two fused silica capillary columns (30 m 0.25 mm) was used to determine retention indices. The operating temperature was set to 35 and then 250°C with a rate of 5°C/minutes, alongside lower and upper temperatures held for 3 and 10 minutes, respectively. The carrier gas (helium) flow rate was 1.0 mL/min. In split mode, a 1.0 L sample was injected (split ratio, 1 : 100). The essential oil constituents were identified by comparing their mass spectra with those of the NIST02 GC/MS library data and the Adams.

### 2.3. Antimicrobial Activity

#### 2.3.1. Antibacterial Activity

Three filamentous fungi, *Aspergillus niger*, *Aspergillus flavus*, and *Fusarium oxysporum*, and one yeast strain *Candida albicans* were used in this study for testing. All fungal strains chosen are pathogenic and belong to drug-resistant microbes. They are among the most contaminating microbes of dried vegetables and cereals and the main producers of mycotoxins. *Candida albicans* is frequently implicated in nosocomial infections. All microbial strains were provided by Sidi Mohamed Ben Abdellah University, Fez, Morocco. Spore suspensions were prepared in a tube containing 0.9% NaCl from seven-day-old cultures on a potato dextrose agar (PDA) medium. The number of spores in suspension was counted using a Malassez cell and the suspensions were diluted to obtain an inoculum concentration of approximately 10^6^ spores/mL [17].

The article "Chemical Characterization and Antioxidant, Antimicrobial, and Insecticidal Properties of Essential Oil from Mentha pulegium L" was published in 2021. Journal: Evid Based Complement Alternat Med.

#### 2.3.2. Antibacterial Activity

In this study, the antibacterial activity of *M. pulegium* EO was tested against four bacterial strains including *Escherichia coli* (ATB: 57) B6N, *Staphylococcus aureus*, *Escherichia coli* (ATB: 97) BGM, and *Bacillus subtilis*. All these strains are pathogenic and provided by Hassan II University Hospital Center's Laboratory of Bacteriology in Fez, Morocco. Müller-Hinton Broth (MHB) and Müller-Hinton Agar (MHA) (provided by VWR Chemicals) were used as growth media for bacteria [1]. Isolated colonies from a fresh culture turn 18h to 24 h were transferred to a 0.9% NaCl solution to prepare the microbial suspension. Next, the optical density of the suspensions was checked with a UV-Visible spectrophotometer at 625 nm and adjusted to be between 0.08 and 0.1 nm, which corresponded to suspensions containing a 10^7^ to 10^8^ CFU/mL according to McFarland [18].

#### 2.3.3. Determination of the Inhibition Zone on Solid Mediums

The disc diffusion technique was used to assess the antibacterial and antifungal activities of *M. pulegium* EO [19]. Briefly, Petri dishes containing BN (nutrient broth) medium were seeded with the tested bacterial strains (*Escherichia coli* (ATB: 57) B6N; *Escherichia coli* (ATB: 97) BGM; *Staphylococcus aureus*; and *Bacillus subtilis*) whilst the MEA (Malt Extract Agar) medium was seeded with *C. albicans*, *A. niger, A. flavus,* and *F. oxysporum.* Next, Whatman paper discs (6 mm in diameter) were placed on the surface of inoculated culture media after being impregnated with 20 *μ*L of EO from *M. pulegium* [20]. After that, the inoculated Petri plates were incubated in the darkness at 30°C for fungal strains and 37°C for bacterial strains, respectively. After 24 hours of incubation for bacterial strains and 48 hours for *C. albicans*, inhibitory diameter and percent inhibition were assessed. After 7 days of incubation, the inhibition diameter and percent inhibition of *A. niger*, *A. flavus,* and *F. oxysporum* were determined [21, 22].

In this study, the negative control was 10 *µ*L of 0.2% agar, whilst fluconazole was used as a positive control with 5 mg/mL in the presence of fungal strains, and streptomycin (0.02 mg/disc) was used as a positive control in the presence of bacterial strains [23].

#### 2.3.4. Determination of Minimum Inhibitory Concentration in the Liquid Medium

The microdilution method was used to determine the lowest inhibitory concentration of *M. pulegium* essential oils against bacterial and fungal strains, according to the method reported by [24]. After 18 hours of incubation for bacteria, 48 hours for yeast, and 7 days for fungi at 30°C [24, 25], the MIC was determined by using the colorimetric method (TTC 0.2% (w/v)) [25, 26].

The article "Chemical Characterization and Antioxidant, Antimicrobial, and Insecticidal Properties of Essential Oil from Mentha pulegium L" was published in 2021. Journal: Evid Based Complement Alternat Med.

### 2.4. Insecticidal Activity

#### 2.4.1. Insect Rearing

The chickpea pest *Callosobruchus maculatus* (*C. maculatus)* was used for insecticidal activity testing. This species was maintained by mass rearing at the laboratory LGME, Department of Chemistry, USMBA, Fez, Morocco. Rearing of *C. maculatus* bruchid was carried out in glass jars with *Cicer arietinum* chickpea seeds. For numerous generations, the jars were kept at a constant temperature of 25°C, relative humidity, and a photoperiod of 14 h (light)/10 h (dark).

#### 2.4.2. Toxicity of Essential Oil against *C. maculatus*

*(1) Assessment of Essential Oil Toxicity by Contact*. Several preliminary tests were conducted to determine the best doses for testing. Afterward, four doses were prepared by dilution including 0.016, 0.079, 0.157, and 0.315 *µ*L/cm^2^, respectively. Filter paper disks with 9 cm diameter (63.62 cm^2^) (Whatman No. 1) were impregnated into EO before being placed in a glass Petri dish of the same diameter, which served to contain the insect. Only acetone was used to treat the disk for the control. In each Petri dish containing 20 g of seeds and a treated washer, a batch of 10 adult insects (5 males and 5 females) were introduced, freshly collected from their rearing environment and no more than 24 hours old (after emergence from seeds). The dishes were then immediately resealed. For each dose, three replicates were used, and dead insects were counted every 24 hours for four days.

In order to calculate the mortality rate, the number of dead insects was counted each day after the experiment ended. Eggs deposited on the walls of boxes and seeds were counted with a binocular loupe to demonstrate the importance of oviposition. The number of eggs of the treated insect was compared to that of the control. The rate of reduction of oviposition was also calculated [26–30].

*(2) Toxicity of EO by Inhalation*. Briefly, a small amount of the cotton was suspended into glass jars. Next, doses of 1 *μ*L, 5 *μ*L, 10 *μ*L, and 20 *μ*L of *M. pulegium* essential oil were deposited into the cotton using a micropipette. Afterward, ten bruchids of *C. maculatus* (male and female) whose ages ranged from 0 and 48 h were placed in each jar and then closed tightly. For each dose, three replications were carried out. The comparison was made with a control sample (cotton without test solutions).

#### 2.4.3. Calculation Methods

The observed mortality rate was corrected by the following formula:

(1) $$\begin{array}{c} Pc=100\times \frac{Po-Pt}{100-Pt}, \end{array}$$

where *Pc* = percent corrected mortality, *Po* = observed mortality in the trial, and *Pt* = observed mortality in the control.

The article "Chemical Characterization and Antioxidant, Antimicrobial, and Insecticidal Properties of Essential Oil from Mentha pulegium L" was published in 2021. Journal: Evid Based Complement Alternat Med.

The following formula was used to calculate the egg-laying reduction rate:

(2) $$\begin{array}{c} Tx=100\times \frac{Nt-Ne}{Nt}, \end{array}$$

where *Tx* = rate of reduction relative to the control, *Nt* = number of eggs in the control jar, and *Ne* = number of eggs in the trial.

### 2.5. Antioxidant Activity

#### 2.5.1. Scavenging of the Free Radical DPPH

In the present study, the protocol used was that described by [31]. Briefly, 0.5 mL of different concentrations of methanol was used to prepare 0.004% DPPH solution. The reaction mixture was stirred immediately before being kept at room temperature (25°C) for 30 minutes in the dark. The absorbance of the reaction medium was measured at 517 nm against a blank containing only methanol. After then, the absorbance was measured and the ascorbic acid was used as a reference. The proportion of DPPH free radical inhibition was estimated using the following method:

(3) $$\begin{array}{c} \%\text{inhibition}=\frac{\text{Abs control}-\text{Abs sample}}{\text{Abs control}}\times 100, \end{array}$$

where Abs control is control absorbance (including all reagents except the test substance) and Abs sample is absorbance of the test compound. The percentage of inhibition was used to calculate the value of IC_50_.

#### 2.5.2. Total Antioxidant Capacity Determination

Three hundred microliters of selected doses of EO was mixed with 3 mL of liquid reactive solution constituted of sulphuric acid, ammonium molybdate, and sodium phosphate. The absorbance was measured using a spectrophotometer set at 695 nm after a 90-minute incubation period at 95°C. The negative control was a blank containing 300 methanol, while the positive control was ascorbic acid [32]. The antioxidant potential of the extracts was measured in mg EAA/g essential oil.

### 2.6. Data Analysis

The results were presented as arithmetic mean values with standard deviation. One-way ANOVA followed by a Tukey test was used to achieve analysis. SPSS version 21.0 was used, and significant values were considered when *P* was less than 0.05.

## 3. Results and Discussion

### 3.1. Extraction Yield and Chemical Composition of Essential Oil

The yield of EO recovered was 2.14 ± 0.22 mL/100 g dry matter. The EO was dried with anhydrous sodium sulfate before being stored in a refrigerator at 4°C until further use. The results of GC/MS analysis of essential oil extracted from *M. pulegium* leaves collected from Ouazzane region are presented in Table 1 and Figure 1. The identified compounds are listed according to the elution order of their retention index.

The article "Chemical Characterization and Antioxidant, Antimicrobial, and Insecticidal Properties of Essential Oil from Mentha pulegium L" was published in 2021. Journal: Evid Based Complement Alternat Med.

The yield of EO from *M. pulegium* leaves was 2.14 ± 0.22 mL/100 g. In this mass, 20 compounds were identified, which represented 98.91% of the total recovered oil. The oil was majority constituted of compounds among R-(+)-pulegone 76.35%, carvone 5.84%, dihydrocarvone 5.09%, and octanol-3 2.25% (Figure 2).

The chemical composition of the studied oils shared some similar compounds with other studies like the pulegone compound [15, 33–35]. The pulegone was also found in EOs from *M. pulegium* belonging to the Mediterranean countries with different proportions.

*M. pulegium* indigenous to Tunisia showed pulegone (61.11%) and isomenthone (17.02%) [36]. *M. pulegium* ingenious to Egypt was found to be also rich in pulegone (43.50%) and piperitone (12.2%) [37]. Environmental factors, the portion of the plant employed, the age of the plant, the phase of the vegetative cycle, and even genetic factors may all play a role in the chemical composition of our sample when compared to that recorded in similar species from other regions [38, 39]. The extraction method can also affect the yield and chemical composition of essential oils, and could therefore, explain the differences in bioactivity [40, 41].

The different biological activities of *M. pulegium* plants were caused by the majority compounds in the essential oils. Pulegone (Figure 2) is the most distinctive chemical of *M. pulegium*, and there are also piperitone (B), menthol (C), menthone (D), and piperitone oxide chemotypes (E) [42, 43]. Furthermore, the EO often contains a high percentage of oxygenated monoterpenes [37], with these chemicals accounting for more than 60% of the total oil [44]. These are known by their activities as biopesticides [45] and the principal contributors to *M. pulegium* EOs' antioxidant activity [46, 47].

(R)-(+)-pulegone is a ketone monoterpene that is found in the essential oils of a variety of plants. It has many bioactivities in cells and animals [48, 49]. According to Damião et al. [50], (R)-(+)-pulegone possessed analgesic therapeutic profile. Roy et al. [51] showed that pulegone reduces LPS-induced inflammation by reducing the effects of NF-*κ*B suggests that pulegone could be used to treat and prevent a variety of inflammatory illnesses. Also, at 40 mM, R-(+)-pulegone reduced *R. dominica* and *L. serricorne* AChE activity by 69.0 percent and 88.0 percent, respectively. Therefore, pulegone can be considered as a good insecticide against these cereal seed pests [52].

### 3.2. Antimicrobial Activity

The antimicrobial activities of EO of *M. pulegium* against pathogenic and phytopathogenic microorganisms were investigated in the present research by the disk diffusion method (Figure 3). The results obtained are presented in Table 2.

The article "Chemical Characterization and Antioxidant, Antimicrobial, and Insecticidal Properties of Essential Oil from Mentha pulegium L" was published in 2021. Journal: Evid Based Complement Alternat Med.

The results showed that the essential oils of *M. pulegium* had a significant inhibitory effect against the tested bacterial and fungal strains. The results indicated that *B. subtilis* was the most sensitive strain tested to *M. pulegium* oil with the highest inhibition diameter (25 ± 0.33). *M. pulegium* oil also showed strong antibacterial activity against *E. coli* (ATB: 57) B6N (10.33 ± 0.44), *E. coli* (ATB: 97) BGM (12 ± 0.66), and *S. aureus* (13.16 ± 0.22). For the antifungal activity, the essential oils of *M. pulegium* also showed an important activity against the tested strains, this activity varied from one strain to another, and the obtained results indicate that *Aspergillus niger* is the most sensitive fungal strain to the oil of *M. pulegium* with a percentage of inhibition up to 100%.

Table 3 shows the MIC findings of *M. pulegium* essential oils against the investigated bacterial and fungal strains. According to the findings, the essential oils of *M. pulegium* have different antibacterial properties. MIC values for bacterial strains (*E. coli* (TBA: 57) B6N, *E. coli* (TBA: 97) BGM, *Staphylococcus aureus*, and *Bacillus subtilis*) ranged from 0.704 to 2.812 g/mL. It can therefore be concluded that low doses of *M. pulegium* oil can inhibit bacterial growth of the tested strains. On the other hand, MIC values for fungal strains (*A. niger*, *A. flavus*, *F. oxysporum*, and *C. albicans*) were between 11.25 and 22.5 *µ*g/mL, which means that the fungal strains tested were more resistant than bacterial strains to essential oils. In addition, the oils of *M. pulegium* showed bactericidal and fungicidal activity against all bacterial and fungal strains tested, respectively. This suggests that the essential oil extracted from *M. pulegium* can be valorized in many fields, especially in food safety thanks to its important antimicrobial activity and its low MIC values against pathogenic and phytopathogenic microorganisms. *M. pulegium* oil has been given high interest to fight resistant bacteria [53]. The essential oils of *M. pulegium* from Ouazzane provide antibacterial effects on a wide spectrum of bacterial strains with different MICs (Gram+: *S. aureus* MBLA: MIC 0.25 mg/mL, *S. Aureus* 976: CMI 1 mg/mL, *S. aureus* 994: CMI 2 mg/mL, *L. monocytogenes*: CMI 0.50 mg/mL; Gram−: *P. Aeruginosa*: CMI 2.00 mg/mL, *Bacillus subtilis*: CMI>2.00 mg/mL, *P. mirabilis*: CMI 0.50 mg/mL, and *Escherichia coli* K12: CMI 0.50 mg/mL) [54]. The essential oils of *M. pulegium* responded differentially to the growth of the bacterial and fungal strains evaluated in our study and elsewhere. In this way, different components may have distinct modes of action, or the metabolism of specific bacteria may be able to counteract the effects of *M. pulegium* oil more effectively. Several studies have shown that the antimicrobial activity of EO can be attributed to its major compounds, such as pulegone (61.10%), isomenthone (17.00%), menthone (5.90%), and piperitone (2.60%) [33], or to the high concentration of piperitone (38%) without excluding any potential synergistic effects of constituents [14].

The article "Chemical Characterization and Antioxidant, Antimicrobial, and Insecticidal Properties of Essential Oil from Mentha pulegium L" was published in 2021. Journal: Evid Based Complement Alternat Med.

*Mentha pulegium* possesses antibacterial effects that are effective against a variety of pathogens for hens [55, 56]. Pulegone, menthone, menthol, and piperitone oxide are responsible compounds for the antibacterial activity of *M. pulegium* [55, 57], while antifungal activity is attributed to aldehydes, alcohols, and ketones (pulegone, menthone, and neo-menthol) [42]. Yeasts are sensitive to EO from *M. pulegium*; however, the effect varies depending on the species and strain [58–60].

### 3.3. Insecticidal Activity

The increasing need for fight-stored chickpea pests has led to an interest in the toxicity of plant-derived EOs. In the present work, we tested the essential oil toxicity at different concentrations against *C. maculatus* for 12, 24, 48, and 72 h. We also calculated LC_50_ values for each EO concentration at the respective treatment times. In this sense, the toxicity of the essential oils was tested by inhalation (Table 4). The 20.0 *µ*L/L air dose showed 100% efficacy against *C. maculatus* after 24 h. Meanwhile, the 5 and 10 *µ*L/L air doses killed all pollution after 72 h. Moreover, all oil concentrations showed more than 70% reduction in oviposition, and more than 90% emergence (Table 5). A total absence of emergence was recorded in batches treated with 10 and 20 *µ*L/mL of EO (Table 6). Previous studies demonstrated EO from closer plant species tested by inhalation against *Sitophilus granarius* (L.) weevils (Coleoptera: Curculionidae); generated 100% mortality after 24 h of treatment with doses of 5, 10, 20, and 40 *µ*L EO/mL acetone [58].

The contact toxicity test showed lower efficacy when compared to the inhalation test; the 20.0 *µ*L/L dose showed 100% mortality after 72 h of exposure. For doses of 5 and 10 *µ*L/L of air, the total mortality was not achieved until beyond 96 h of exposure. The lethal dose of the 24-hour inhalation test LC_50_ was 1.99 mL/L air, with a 95% confidence interval (0.27–4.127) over 48 h was 0.83 mL/L air (Table 7). For the contact test, the LC_50_ was 6.51 mL/L of air over 24 h of exposure; this value became lower after 48 and 72 h of exposure (Table 8). It is thus fitting that EOs of *M. pulegium* tested by inhalation can be a promising source of active compounds to fight chickpea pests. The 20.0 mL/L dose was the most active and could be an interesting ecological alternative to eliminate *C. maculatus* from stored seeds.

The article "Chemical Characterization and Antioxidant, Antimicrobial, and Insecticidal Properties of Essential Oil from Mentha pulegium L" was published in 2021. Journal: Evid Based Complement Alternat Med.

The insecticidal activity of *M. pulegium* oil has been tested against some insects in previous studies. These studies were mainly classified according to the life stage of the target insect (i.e., adult, larva, and other closer species). Our results showed that *M. pulegium* EOs exhibited efficacy against *Callosobruchus maculatus*. These results are in agreement with those reported in earlier work [12, 13, 15, 58, 61].

The chemical composition of *M. pulegium* oil, in general, and the monoterpenes that function as insecticidal agents in particular, are responsible for its efficiency [62–64]. Monoterpenes, particularly pulegone, are abundant in our plant (76.35 percent). These active ingredients had significant insecticidal efficacy against a variety of pests [62, 65]. Pulegone has the ability to enter the lipophilic cuticular tissue layer of insects, resulting in the suppression of respiration, growth, and fecundity. The mechanism of action of the responsible compound can also include the acetylcholinesterase inhibition [66, 67]. Interference with octamine action, gamma-aminobutyric acid (GABA), modulation of chlorine channels has also been reported in previous works [68, 69]. In addition, it should be noted that the method of application (inhalation or contact) of *M. pulegium* EO on *C. maculatus* showed differences in the percentage of mortality, fecundity rate, and emergence rate.

### 3.4. DPPH Free Radical Scavenging

The DPPH bioassay was used to assess the antiradical activity of *M. pulegium* essential oils. Ascorbic acid (vitamin C) was employed as a standard reference to attain this purpose.  Figure 4 depicts the antiradical action of *M. pulegium* essential oil. The essential oils of *M. pulegium* had an IC_50_ of 7.659 mg/Ml for antioxidant activity against the DPPH radical. This finding is consistent with prior research, which found that oil from *M. pulegium*, a native of Iran, had an antioxidant activity with an IC_50_ of 14736 g/mL [11]. When compared to the standard synthetic antioxidant (Figure 5), ascorbic acid (IC_50_ = 2.815 *µ*g mL) (P0.0001), these essential oils have a moderate antioxidant potential. The chemical composition of *M. pulegium* essential oils accounts for their antioxidant action [70]. Pulegone (61.11%) may be implicated in *M. pulegium's* antioxidant action [70]. The obtained results are supported by those reported elsewhere, which showed that essential oil from *M. pulegium* from different collection areas had antioxidant power [36].

The article "Chemical Characterization and Antioxidant, Antimicrobial, and Insecticidal Properties of Essential Oil from Mentha pulegium L" was published in 2021. Journal: Evid Based Complement Alternat Med.

### 3.5. Total Antioxidant Capacity (TAC)

The measurement of the total antioxidant capacity revealed the presence of important antioxidant agents in the studied oil (583.066 ± 57.05 mg EAA/g EO) (Figure 4). Our results were in agreement with those reported by Ahmed et al. [7], who showed antioxidant activity (IC_50_ = 20.17 ± 1.88 mg/mL) in essential oils from *M. pulegium* collected from the different collection areas. In addition, the same authors reported that the studied EOs were potent when compared to reference antioxidants, butylated hydroxytoluene (BHT).

Ahmed et al. [7] discovered that the modest variations in components, mainly pulegone and menthone concentrations, can be attributable to the varying degrees of antioxidant capabilities found for EOs isolated from *M. pulegium* dried by different procedures. In this sense, it was reported that pulegone and menthone identified in *M. pulegium* may be the responsible compounds for the antioxidant effect [11, 62–73].

The active molecules in essential oils of aromatic plants are primarily responsible for their antioxidant properties, according to the literature. The monoterpene ketones menthone and isomenthone are the most powerful molecules [74]. Minor molecules in essential oils, rather than large compounds, are more likely to have a substantial role in antioxidant activity [75]. Similarly, previous works showed the presence of very important antioxidant activity of several essential oils including genus *Mentha* essential oil [76].

## 4. Conclusion

The chemical composition and antioxidant, antibacterial, and insecticidal activities of *M. pulegium* L. were studied in this work. In conclusion, the essential oil of *M. pulegium* L. was found to be very rich in R-(+)-pulegone, which remains the main contributor to the biological activities of this oil. This study revealed that the essential oil of *M. pulegium* was active against the tested microbes, insect pests of legume seeds along with antioxidant effect so that the plant oil can be used as natural drugs to serve health and food crops. Therefore, the essential oil of *M. pulegium* can be exploited in the development of antibiotics, bioinsecticides, and food preservatives. However, on a large-scale practical level, it is necessary to better understand the effect of sublethal doses of essential oils on nontarget organisms, as well as potential toxicities to humans. It is thus fitting that further studies on the potential toxicities of the tested essential oils are needed for safety purposes.

The article "Chemical Characterization and Antioxidant, Antimicrobial, and Insecticidal Properties of Essential Oil from Mentha pulegium L" was published in 2021. Journal: Evid Based Complement Alternat Med.

## Figures and Tables

**Figure 1:** Chromatogram of essential oil from *M. pulegium* leaves.

**Figure 2:** Chemical structure of the main compounds of *M. pulegium* EO determined by the ChemBioDraw software (Ultra 11.0).

**Figure 3:** Pictures showing the antifungal and antibacterial activities of the studied essential oils. (a) Antifungal activity; (b) negative control for antifungal activity; (c) antibacterial activity; (d) negative control for antibacterial activity.

**Figure 4:** Results of the DPPH antioxidant test for *Mentha pulegium* essential oils.

**Figure 5:** Results of the antioxidant test by the DPPH method for ascorbic acid.

**Table 1:** Constituents of the essential oil of *M. pulegium* identified by GC-MS analysis.

Compounds	Components	RI	Area (%)
1	*α*-Pinene	937	0.69
2	Cyclohexanone-3-methyl	952	0.37
3	*β*-Pinene	974	0.52
4	Myrcene	992	0.14
5	Octanol-3	995	2.25
6	D-2-Carene	1003	Tr
7	Limonene	1030	1.41
8	*p*-Mentha-3.8-diene	1071	1.95
9	Menthone	1150	0.08
10	Pinocarvone	1166	1.76
11	Isomenthol	1182	0.28
12	Menthol	1171	0.62
13	Dihydrocarvone	1193	5.09
14	R-(+)-pulegone	1236	76.35
15	Carvone	1240	5.84
16	*α*-Peperitone	1251	0.36
17	Caryophyllene	1418	0.18
18	Germacrene D	1475	0.09
19	*γ*-Eudesmol	1630	0.37
20	*α*-Eudesmol	1649	0.56
Total identified			98.91

**Table 2:** Antibacterial and antifungal effect of *Mentha pulegium* EOs against bacterial fungal strains.

Antibacterial activity (inhibition diameter in mm)			Antifungal activity (percentage of inhibition)		
Bacterial strains	EOs	SPM	Fungal strains	EOs	FLU
*E. coli (ATB:*57)	10.33 ± 0.44	—	*A. niger*	100 ± 0.00%	89.75 ± 0.41%
*E. coli (ATB:*97)	12 ± 0.66	—	*A. flavus*	87.91 ± 0.08%	94.42 ± 0.92%
*S. aureus*	13.16 ± 0.22	9.73 ± 0.23	*F. oxysporum*	92.91 ± 0.09%	91.91 ± 0.9%
*B. subtills*	25 ± 0.33	10.52 ± 0.41	*C. albicans*	23 ± 0.66 %	95.81 ± 0.76%

EOs: essential oils of *Mentha pulegium*; SPM: streptomycin; FLU: fluconazole; and (−): non-inhibition.

**Table 3:** Minimal inhibitory concentration of *Mentha pulegium* essential oils against the four bacterial and four fungal strains.

Antibacterial activity		Antifungal activity	
Bacterial strains	Minimal inhibitory concentration (MIC) (*µ*g/mL)	Fungal strains	Minimal inhibitory concentration (CMI) (*µ*g/mL)
*E. coli (ATB:*57)	0.704	*A. niger*	11.25
*E. coli (ATB:*97)	1.406	*A. flavus*	22.5
*S. aureus*	1.406	*F. oxysporum*	22.5
*B. subtills*	2.812	*C. albicans*	11.25

**Table 4:** Effects of essential oils of *M. pulegium* tested by inhalation on the mortality of *C. maculatus*.

Dose (*µ*m)	Percentage of mortality per treatment day			
	24 h	48 h	72 h	96 h
Control	0 ± 0^a^	0 ± 0^a^	0 ± 0^a^	0 ± 0^a^
1	43.3 ± 4.4^b^	63.3 ± 5.7^b^	86.7 ± 5.7^b^	93.3 ± 11.5^b^
5	63.3 ± 4.4^c^	73.3 ± 5.7^b^	100 ± 0^c^	100 ± 0^c^
10	80 ± 6.6^d^	90 ± 10^c^	100 ± 0^c^	100 ± 0^c^
20	100 ± 0^e^	100 ± 0^c^	100 ± 0^c^	100 ± 0^c^

Columns with the same letter did not differ significantly according to ANOVA analysis.

The article "Chemical Characterization and Antioxidant, Antimicrobial, and Insecticidal Properties of Essential Oil from Mentha pulegium L" was published in 2021. Journal: Evid Based Complement Alternat Med.

**Table 5:** Effects of essential oils from *M. pulegium* tested by contact on oviposition and emergence of *C. maculatus*.

Dose (*µ*m)	Number of eggs and emergence	
Number of eggs laid emergence	Number of eggs adults emergence
Control	0^a^	0^a^
1	74.64 ± 21.2^b^	13.67 ± 2.51^b^
5	83 ± 1.86 ^bc^	6.33 ± 1.84^b^
10	98.33 ± 0.41^c^	100 ± 0^b^
20	100 ± 0^c^	100 ± 0^b^

Columns with the same letter did not differ significantly according to ANOVA analysis.

**Table 6:** Lethal concentration values of *M. pulegium* essential oil tested by inhalation on *C. maculatus*.

Treatment (h)	df	Slope + SD	LC_50_ (CI95%)	LC_95_ (CI95%)	Intercept ± SE	*p* value	*X* ^2^
24	2	1.41 + 0.48	1.99 (0.27;4.127)	28.81 (10.93;1900.8)	−0.424 + 0.382	0.409	1.79
48	2	1.17 + 0.51	0.83 (0.0;2.298)	20.8 (7.03; 661438)	0.96 + 0.379	0.430	1.69
72	2	—	—	—	—	—	
96	2	—	—	—	—	—	—

(—): data are absent because the insects died within the first hour of the experiment.

**Table 7:** Effects of essential oils of *M. pulegium* tested by contact on the mortality of adults from *C. maculatus*.

Dose (*µ*m)	Percentage of mortality per treatment day			
	24 h	48 h	72 h	96 h
Control	0 ± 0^a^	0 ± 0^a^	0 ± 0^a^	0 ± 0^a^
1	16.67 ± 4.44^b^	33.33 ± 4.44^b^	53.33 ± 4.44^b^	90 ± 0^b^
5	26.67 ± 4.44^b^	53.33 ± 4.44^c^	76.67 ± 4.44^c^	100 ± 0^b^
10	60 ± 6.67^c^	73.33 ± 4.44^d^	93.33 ± 4.44^d^	100 ± 0^b^
20	86.67 ± 4.44^d^	96.67 ± 4.44^e^	100 ± 0^d^	100 ± 0^b^

Columns with the same letter did not differ significantly according to ANOVA analysis.

**Table 8:** Lethal concentration values of *M. pulegium* essential oil tested by contact on *C. maculatus*.

Treatment (h)	df	Slope + SD	LC_50_ (CI95%)	LC_95_ (CI95%)	Intercept ± SE	*p* value	*X* ^2^
24	2	1.56 ± 0.5	6.51 (2.95; 15.06)	74.18 (25.2; 5759.5)	−1.268 + 0.457	0.004	2.01
48	2	1.38 ± 0.51	2.74 (0.53; 0.69)	42.71 (14.9; 4580.6)	−0.603 + 0.389	0.002	2.009
72	2	1.47 ± 0.55	1.026 (0.032; 2.34)	13.43 (5.58; 806.95)	−0.017 ± 0.381	0.007	0.832
96	2	—	—	—	—	—	—

(—): data is absent because the insects died within the first hour of the experiment.

## Data Availability

Data used to support the findings are included within the article.
